This article has been retracted.

# Combination therapy with Nab-paclitaxel and the interleukin-15 fused with anti-human serum albumin nanobody as a synergistic treatment for colorectal cancer

**DOI:** 10.1080/21655979.2021.2023997

**Published:** 2022-01-12

**Authors:** Lipei Wu, Weiwei Wang, Jiale Tian, Chunrun Qi, Zhengxin Cai, Wenhui Yan, Shihai Xuan, Anquan Shang

**Affiliations:** a Department of Laboratory Medicine, Dongtai People’s Hospital & Dongtai Hospital of Nantong University, Yancheng, China; b Department of Laboratory Medicine, Shanghai Tongji Hospital, Shanghai, China; c Department of Pathology, Tinghu People’s Hospital, Yancheng, China; d Department of Laboratory Medicine, Tinghu People’s Hospital of Yancheng City, Yancheng, China

**Keywords:** Nab-paclitaxel, IL-15, anti-HSA nanobody, synergistic treatment, colorectal cancer

## Abstract

This study determines the effect of Nab-paclitaxel in combination with IL-15 fusion protein, containing IL-15 and an anti-HSA nanobody domain, on colorectal cancer bearing mice. *In vitro* binding test of IL15 fusion protein to HSA and Nab-paclitaxel, as well as CTLL-2 cell stimulation assay were performed. The tumor inhibitory effects of Nab-paclitaxel in combination with IL-15 fusion protein was evaluated in the HCT116 bearing murine model. Moreover, the population and function of cytotoxic T cells and M1 macrophages, as well as MDSCs and Treg cells, were also further examined. As a result, combination therapy of Nab-paclitaxel and IL-15 fusion protein effectively inhibits the tumor growth and produced a 78% reduction in tumor size for HCT116, as compared to vehicle group. In the TDLN for the combination group, there were 18% of CD8+ IFN-γ + T-cells and 0.47% CD4^+^CD25^+^FOXP3^+^ regulatory T-cells, as opposed to 5.0% and 5.1%, respectively, for the model control group. Combination therapy further exhibited enhanced suppressive effects on the accumulation of CD11b^+^GR-1^+^ MDSC in spleen and bone marrow. Furthermore, Nab-paclitaxel and IL-15 fusion protein showed a significant suppression of NF-κB-mediated immune suppressive markers and increased expression of CD8, Granzyme B, CD62L, CD49b, and CD86 without obvious organ toxicity. In conclusion, combination therapy of Nab-paclitaxel and IL-15 fusion protein can effectively stimulate the antitumor activity of immune effector cells, thereby inhibiting immunosuppressive cells within the TME of colorectal cancer, and the overall therapeutic effect has a significant advantage over monotherapy.

Abbreviations

Interleukin 15, IL-15; Human serum albumin, HSA; Myeloid-derived suppressor cells, MDSC; Albumin binding domain, ABD; Tumor drainage lymph node, TDLN; Natural killer (NK); Tumor-draining lymph node (TDLN); Tumor infiltrating lymphocyte, TIL; Immunogenic cell death, ICD; Enhanced permeability retention, EPR; Liposomal doxorubicin, Doxil; 5-fluorouracil, 5-FU.

## 1. Introduction

Colorectal cancer is one of the most significant medical challenges and has a very poor 5-year survival rate [1,2]. The poor prognosis for colorectal cancer is mainly due to the difficulty of making an early diagnosis, resistance to therapies and a high probability of tumor recurrence after treatments [3,4]. 5-FU monotherapy has been a standard chemotherapy for colorectal patients since its approval, but in the following period of more than a decade, numerous clinical trials combining 5-FU with other chemotherapies failed to demonstrate significant advantage due to toxicity [5,6].

Nab-paclitaxel is a paclitaxel in the albumin-bound form of nanoparticles, which has a mean particle size of 120–130 nm [7]. In terms of clinical application, the FDA has approved its use in patients with metastatic breast cancer who fail to respond to combination chemotherapy or relapse within 6 months after adjuvant chemotherapy [8,9]. In a clinical trial for the treatment of metastatic colorectal cancer, Nab-paclitaxel combined with gemcitabine significantly prolonged the response rate, progression-free survival, and overall survival of patients relative to monotherapy [10].

In addition to conventional treatments, including surgical resection, radiotherapy, and chemotherapy, the use of the patient’s own immune system to inhibit the occurrence and development of tumors is currently the focus of immunotherapy anticancer [11,12]. For example, immune checkpoint inhibitors currently approved by the FDA for marketing, including monoclonal antibodies against PD-1 or CTLA-4, have been successfully applied in the clinical treatment of a variety of cancers [13–15]. However, immunotherapy has no significant inhibitory effect on colorectal cancer, which is mainly due to immune escape and the inability of effector cells of the immune system to effectively enter the tumor microenvironment, specifically manifested as dense fibrotic tissue, scarce cytotoxic T lymphocytes, and natural killer cells, as well as upregulated regulatory T cells and myelogenous suppressor cells, which together cause immunosuppression, thus making colorectal cancer refractory [2]. In addition, upregulation of NF-κB expression may form an immunosuppressive tumor microenvironment in various types of cancer. Therefore, current therapies categorize colorectal cancer as a ‘cold’ tumor [16].

IL-15 is a potent immune stimulator that is critical for the proliferation and activation of NK and CD8^+^ T cells [17]. By acting on T cells, IL-15 stimulates their proliferation and allows them to secrete cytokines that kill tumor cells, such as IFN-γ and TNF-α, which show a variety of biological activities and exert their antitumor effects, making ‘cold’ tumors ‘hot’ [17]. A novel long-acting IL-15, including an anti-HSA nanobody and a human IL-15, were designed and prepared. Previous data demonstrated the similar in vitro activity and enhanced in vivo stability compared with wild type IL-15 [17]. In current study, we hypothesized that complementary strategies of combined chemotherapy and with immunotherapy may be effective against colon cancer. Hence, we investigate the protective effect of combination therapy with IL-15 fusion protein and Nab-paclitaxel on colon tumor in rodent animals.

## 2. Materials and methods

### 2.1 Materials

Flow cytometry related antibodies, such as CD4, CD8, CD11b, CD25, CD86, Foxp3, Gr-1, IFN-γ were all purchased from BD Pharmingen (San Diego, CA, USA). IHC related antibodies, including CD8 (Sino Biological, Beijing, China), CD86 (Cell Signaling Technology, Danvers, MA, USA), NF-κB (ser536), Cleaved caspase-3, -8, -9 (Cell Signaling Technology), Foxp3 (Elabscience), Granzyme B, IDO (Sigma Aldrich, Louis, MO, USA) Ki-67, and VEGF (Elabscience) were purchased from indicated companies. Nab-paclitaxel was purchased from Taipei Veterans General Hospital Pharmacy.

### 2.2 Plasmid construction and protein preparation

In brief, the gene of IL-15 fused anti-HSA Nanobody was prepared via gene synthesis and then cloned into the commercial pcDNA3.1 plasmid vector. The final sequence of construct was confirmed by DNA sequencing. Human embryonic kidney 293 (HEK293) cells were transfected with the correctly sequenced recombinant vectors by lipofectin according to conventional methods. Then the supernatants of transfected cell were collected and concentrated by Amicon® Ultra 10 kDa centrifugal filters (EMDMillipore, Germany). The concentrated supernatant was purified by affinity chromatography. Finally, the purified samples were buffered exchange by dialysis against 2 L of PBS at 4°C for 20 h. The biochemical characterization of IL-15 fusion protein, including were further performed via SDS-PAGE gel and HPLC-SEC analysis (data not shown) with purity over 95%.

### 2.3 Cell culture

HCT116 cells and CTLL-2 murine T-cell lines were brought from ATCC. The CTLL-2 cells were cultured in RPMI 1640 supplementing with 10% FBS, 2 mM Glutamine and 150 IU/mL IL-2. The HCT116 cells were cultured in RPMI 1640 medium and DMEM, supplemented with 10% FBS, 90 units/mL penicillin, 3 mM l glutamine, and 90 μg/ml streptomycin (5% CO_2_ at 37°C).

### 2.4 In vitro binding test

HSA and Nab-paclitaxel were immobilized on a 96-well plate and then blocked with 5% BSA, followed by washing three times with PBST. IL-15 fusion proteins were performed gradient dilution and then incubated with HSA or Nab-paclitaxel, followed by washing with PBST. Further detection was performed via HRP-tagged antibody and TMB substrate, and then inhibited by ELISA stop solution. Further results were obtained at 450 nm via applying the plate reader.

### 2.5 The stimulation of CTLL-2 cells by HCT116-luc cells treated with Nab-paclitaxel and IL-15 fusion protein

The phosphorylation of STAT-5 was detected to assess the activation of CTLL-2 cells, which were co-cultured with HCT116-luc cells that pre-treated with Nab-paclitaxel and IL-15 fusion protein via using flow cytometry. In brief, the HCT116-luc cells at the concentration of 3*10^4^ cells/well were incubated with the Nab-paclitaxel and IL-15 fusion protein at the final concentration of 0, 100, 300, and 1000 nM and 0, 100, 300, and 1000 ng/mL, respectively. The fixed cells were subjected to permeabilization, rehydration and incubation with antibody targeting phosphorylated-STAT5 and then treated with secondary antibody and then detected by using flow cytometer.

### 2.6 Animal experiments

Animal experiments were approved by the Animal Care and Use Committee. The C57BL/6 mice (female, 6–8 weeks) were obtained and the kept in a pathogen-free facility. HCT116 cells (2x10^5^ cells/mouse) were inoculated in the right flank of mice. After 7-day, the mice were assigned into 4 groups: a vehicle control (n = 5), Nab-paclitaxel (300 μg, n = 6), IL-15 fusion protein (10 μg, n = 6) and combined treatment of Nab-paclitaxel and IL-15 fusion protein (n = 6), when the tumor grow to about 110 mm^3^. Tumor volume was assessed via a caliper and calculated as follows: Tumor volume = tumor length × tumor width^2^ × 0.523 [17].

The protocols for the IHC staining were referred to the previous reports [18]. Staining slices were acquired at 200 × magnification. Quantification results for protein expression on IHC slides were analyzed using ImageJ software.

Immune profiling of TILs, TDLN, spleen and bone marrow with flow cytometry. In brief, the CD4^+^, CD8^+^ T cells, M1 macrophages, Tregs cells and MDSCs in bone marrow, TDLN and TIL were determined via flow cytometry according to the previously reported methods [19].

### 2.7 Statistical analysis

All data were presented as mean ± SEM. One-way ANOVA method was applied to analyze the difference by using GraphPad Prism 8.4. The *p* value < 0.05 was considered as the significant difference.

## 3. Results

In current study, we hypothesized that complementary strategies of combined chemotherapy and with immunotherapy may be effective against colon cancer. Hence, we investigate the protective effect of combination therapy with IL-15 fusion protein and Nab-paclitaxel on colon tumor in rodent animals. In vitro study revealed that IL-15 fusion protein couples to Nab-paclitaxel with a high affinity and may form a bifunctional nanotherapeutic that stimulates immunity and cytotoxicity. Furthermore, current research also demonstrated the combined effects of IL-15 fusion protein with Nab-paclitaxel on colon cancer subcutaneous HCT116 model.

### 3.1 IL-15 fusion protein coupled to Nab-paclitaxel on cancer cells

As the results shown in Figure 1(a), similar binding affinities of IL-15 fusion protein for HSA and Nab-paclitaxel at 10.5 and 12.5 nM, respectively, were observed. Moreover, the binding of IL-15 fusion protein binding to HSA or Nab-paclitaxel was suppressed by adscititious HSA in a dose-dependent manner (Figure 1(b)). The uptakes of IL-15 fusion protein by either murine cancer cells in the presence or absence of Nab-paclitaxel were further assessed. As the results showed in Figure 1(c), IL-15 fusion protein exhibited similar Nab-paclitaxel uptakes by HCT116 cells.

**Figure 1.** *In vitro* studies of IL-15 fusion protein, Nab-paclitaxel alone or combination. (a) Binding test. (b) Competition test. (c) IL-15 fusion protein uptakes test. (d) STAT-5 phosphorylation of Nab-paclitaxel and (e) IL-15 fusion protein group. All data were presented as mean ±SEM (n = 3). *p < 0.05, ** *p* < 0.01, and ***p < 0.001.

### 3.2 IL-15 fusion protein coupled to Nab-paclitaxel enhance immune activation

In order to determine whether the IL-15 fusion protein coupled to Nab-paclitaxel reserve the ability to regulate immunity, the CTLL-2 cells were further coincubated with HCT116 cells and two molecules, and the phosphorylated STAT-5 was measured. As the results showed in Figures D-E, significantly activated STAT-5 phosphorylation were observed when CTLL-2 cells were cocultured with Nab-paclitaxel and IL-15 fusion protein within the ranges of 300 and 1000 nM, 300 and 1000 ng/mL, respectively.

### 3.3 IL-15 fusion protein enhanced antitumor efficacy of Nab-paclitaxel in HCT116 cells murine models

HCT116 cells bearing xenograft model were used to assess the treatment efficacy of IL-15 fusion protein and Nab-paclitaxel alone or combination. As shown in Figure 2(a), model mice received the saline, IL-15 fusion protein, Nab-paclitaxel alone or combination 2 per week for 2 weeks by intravenous injection. As the results showed in Figure 2(b), the tumor does not progress as quickly for the combination group as for each single treatment, while the combination therapy exhibited enhanced tumor growth inhibition. Moreover, the mean tumor weight for the combination group is significantly lower than those of two mono-treatment groups (Figure 2(c)).

**Figure 2.** Anti-tumor test in HCT116 models. (a) Study design in HCT116 xenograft animal model. (b) Tumor growth-time curve. (c) Tumor weight. (d) Ki-67 expression data. (e) Body weight and (f) change of HCT116 xenograft mice. All the results were showed as Mean ± S.E.M, n = 6. a1, a2 vs. control *p* < 0.05, *p* < 0.01; b2 vs. Nab-paclitaxel. *p* < 0.01; c2 vs. IL-15 fusion protein *p* < 0.01).

In order to further determine the antitumor effects of combined treatment. The expression level of Ki-67, a proliferation marker, was determined using IHC, and results showed lower expression in xenograft HCT116 received the treatment of combo than those of others (Figure 2(d)), demonstrating that that IL-15 fusion protein sensitizes HCT116 to Nab-paclitaxel.

Moreover, the effective dose of Nab-paclitaxel combined with IL-15 fusion protein does not induce a pathological change in normal organs tumor-bearing mice. As evidence showed in Figure 2(e,f), the body weight of subcutaneous HCT116-bearing mice showed no statistically significant difference between groups. Furthermore, the general condition and liver function of experimental mice was not affected by Nab-paclitaxel, IL-15 fusion protein or a combination of both (data not shown).

### 3.4 Nab-paclitaxel combined with IL-15 fusion protein potentiated anticancer immunity in murine cancer models

In order to determine the systemic and local immune activation induced by combination therapy, analysis of immune population within mice spleen, BM, TDLNs, and TILs were conducted. As the results showed in Figure 3a, the CD4^+^ T cells, representing the population of memory T cells, was significantly increased for the group received combined treatment. Similar change was observed in the CD8^+^ T cells, as the cytotoxic T cells population (Figure 3(b)). Moreover, the populations of CD11b^+^CD86^+^ M1^−^like macrophages in BM and TIL were also significantly increased in the combination therapy group (Figure 3(c,d)). As showed in Figure 3(e), the population of CD8^+^ T cells increased from 26.2% to 60.1% after combination therapy. Meanwhile, the population of CD8^+^ T cells in TDLN was also increased by the combination treatment (Figure 3(g)). The activation of IFN-γ of CD8^+^ T cells in TIL or TDLN increased 12-fold or 4-fold in combination group than that of the control group, respectively (Figure 3(f,h)).

**Figure 3.** Effects of combination therapy on population and function of cytotoxic T cells and M1 macrophage. Quantification results of (a) CD4 + T cells in TDLN and (b) CD8^+^ T cells in SP, (c) CD8^+^ T cells and (d) CD8^+^ IFN-γ^+^ T cells in TDLN, (e) CD8^+^ T cells and (f) CD8^+^ IFN-γ^+^ T cells from TILs, (g) CD11b+CD86+ M1-like macrophage in BM and (h) CD11b^+^CD86^+^ M1-like macrophage in BM from TIL. (i) Quantification results of CD8, Granzyme B, CD62L, CD49b, and CD86. All the results were showed as Mean ± S.E.M, n = 6. a1, a2 vs. control p < 0.05, p < 0.01; b2 vs. Nab-paclitaxel *p* < 0.01; c2 vs. IL-15 fusion protein *p* < 0.01.

The expression level of various markers of immune activation, including CD8, granzyme B, CD62L, CD49b and CD86 in tumor tissues were further detected (Figure 3(i-j)). CD8 and Granzyme levels were increased in the group received combination therapy. Similarly, the memory T cell and NK cell markers, including CD62L and CD49b were also increased. Moreover, the CD86 expression was significantly induced by IL-15 fusion protein and Nab-paclitaxel combination, consistent with the flow cytometry data displaying accumulation of CD11b^+^CD86^+^ M1-like macrophages within tumors from mice of combination group. Above data collectively suggested that the Nab-paclitaxel marginally increases accumulation of CD8 cells M1-like macrophage as well as cytotoxicity in the systemic and local immune systems.

### 3.5 Nab-paclitaxel combined with IL-15 fusion protein attenuated the NF-κB mediated immunosuppressive effect and enhanced apoptosis signaling murine cancer models

As the results showed in Figure 4(a,b), the significantly decreased NF-κB phosphorylation was observed in the group received the combined treatment. The MDSC presenting in BM and spleen of HCT116 tumor tissues were evaluated to assess the effect of combined treatment on immunosuppressive cells. Results were showed in Figure 4(c,d), MDSCs in BM and spleen were significantly reduced after the combined treatment, compared to the control group. Moreover, the Foxp3 was significantly suppressed in TDLN of mice received the combination therapy (Figure 4(e)). Similar results were showed in the expression levels of other immune suppressive factors, such as IDO and VEGF, which all exhibited significantly decrease induced by the combination therapy. These results collectively demonstrated that combined treatment inhibited the immunosuppression. In order to determine whether the apoptosis signaling pathway is also activated by combined treatment, the protein expression levels of cleaved caspase-3, -8, and -9 in tumor tissues was assessed. As the results showed in Figure 5, the protein expression level of cleaved caspase-3 was 2.3-folds greater in the combination group than the control group. There was also 2.0-fold higher expression level of extrinsic apoptosis marker, cleaved caspase-8, in the combination group (Figure 5(b)). The protein expression of cleaved caspase-9 involved in the intrinsic apoptosis pathway, was triggered by combination therapy. The level of expressed apoptotic protein that was greater for the combination treatment for the xenograft animal models.

**Figure 4.** Effects of combination therapy on population and function of Treg cells and MDSCs. (a) Quantification results of NF-κB (ser536). Quantification results of MDSCs in (b) BM and in (c) SP, and (d) CD4+ CD25+ Foxp3+ Treg in TDLN. All the results were showed as Mean ± S.E.M, n = 6. a1, a2 vs. control *p* < 0.05, *p* < 0.01; b1, b2 vs. Nab-paclitaxel *p* < 0.05, p < 0.01; c1, c2 vs. IL-15 fusion protein *p* < 0.05, *p* < 0.01.

**Figure 5.** Effects of combination therapy on extrinsic and intrinsic apoptotic pathway. Quantification results of (a) CD11b, Gr-1, Foxp3, IDO and VEGF, and (b) cleaved caspase-3, -8, and -9. All the results were showed as Mean ± S.E.M, n = 6. a1, a2 vs. control *p* < 0.05, *p* < 0.01; b1, b2 vs. Nab-paclitaxel *p* < 0.05, *p* < 0.01; c1, c2 vs. IL-15 fusion protein *p* < 0.05, *p* < 0.01.

## 4. Discussion

Nab-paclitaxel is a unique nanoparticle of an albumin-bound form of paclitaxel, which has a higher response rate and enhanced safety profiles, compared with a solvent-based formulation of paclitaxel [8]. Nab-paclitaxel is associated with a prolonged half-life, increased accumulation in the tumor, macropinocytosis-driven activation of macrophages, apoptosis of cancer cells and improved accessibility for immune cells and therapeutics to the TME through stromal depletion [20]. However, the prognosis for colon cancer patients is very poor and this remains a significant challenge [21].

Colon cancer is relatively resistant to chemotherapy or immunotherapy because the tumor is surrounded by an extracellular fibrotic barrier that is formed by collagen, fibronectin and hyaluronic acid, which prevents the delivery of sufficient chemodrugs and infiltration of the immune effector cells [22,23]. The lack of NK and CD8 + T cells within the TME characterizes colon cancer as a cold tumor so there may be a beneficial effect for immune stimulants that are combined with chemotherapy, so that is challenged by toxic drug becomes a hot tumor when it is infiltrated by active immune effector cells [17,24]. In addition to tumor cells, which are the major target of conventional anticancer therapy, stromal, endothelial and immune cells all play a critical role in the progression, survival and metastasis of tumor cells [13].

Nanomedicine is an increasingly common strategy for targeting TME with multiple complementary therapeutic, including cytotoxic drugs, radiation and immunotherapy [25]. Doxil and Nab-paclitaxel, which have an average respective size of around 150 and 130 nm, are some of the first nanoparticle chemotherapies in clinical use [26]. Their size allows improved tumor localization and a better safety profile because of EPR [26]. As opposed to the normal organs, tumor is often associated with disorganized blood vessels and there is no tight junction between endothelial cells [27]. Some chemodrugs, such as doxorubicin and paclitaxel, which are major components of Doxil and Nab-paclitaxel, respectively, can trigger ICD within the TME, but chemodrug-induced anticancer immunity has not been frequently demonstrated for long term tumor suppression [26]. The multiple key steps in the cancer-immunity cycle mean that a combination of complementary therapeutics may affect different immune regulatory steps, such as tumor killing, antigen release, processing, presentation, activation, and infiltration of immune effect cells and inhibition of the immune checkpoint [28].

IL-15 is one of the type I family members of IL2 [29]. It supports the proliferation, activation and survival of NK and CD8^+^ T cells in the absence of Treg activation and has no role in AICD [29]. Given its positive effects on anticancer immunity, IL-15 was ranked as the most promising immunotherapy for cancer treatment by an immunologist panel at a National Cancer Institute workshop [30]. In the first dose-escalating clinical trial, IL-15 was intravenously administered for 12 consecutive days to patients with metastatic renal cell carcinoma and melanoma and its efficacy is evident in some patients with clearance of metastatic lesions [31]. Clinical studies demonstrate that N-803 in combination with the anti-PD-1 monoclonal antibody, nivolumab, gives good results in trial for patients with refractory metastatic nonsmall cell lung cancer [32].

In current we used the hIL-15 fusion protein, which is composed of hIL-15 fused with an anti-HSA nanobody to preserve the immune stimulating effect of hIL-15 and the high binding affinity to albumin to give a prolonged half-life in experimental mice. The tumor suppressing activity of IL-15 fusion protein is correlated with the activation of NK cells and CD8^+^ T cells and a decrease in MDSCs and Tregs within the TME. Overexpression of NF-κB may trigger immunosuppressive cascades to develop immunosuppressive TME, and we hypothesized that the phosphorylation of NF-κB was effectively suppressed by Nab-paclitaxel combined with IL-15 fusion protein.

In current study, IL-15 fusion protein was demonstrated with potent albumin binding capability and couples to Nab-paclitaxel in nanoparticle form, which is composed of human albumin and paclitaxel in a ratio of 9:1. Our in vitro study showed that IL-15 fusion protein couples to both HSA and Nab-paclitaxel with a similar affinity (Figure 1(a)), indicating this complex could form a bifunctional nanotherapeutic that stimulates immunity and cytotoxicity. The binding affinity of IL-15 fusion protein and Nab-paclitaxel contributes to the superior effect of the combination, which may exhibits better anticancer activity. Current study exhibited that IL-15 fusion protein combined with Nab-paclitaxel could stimulate the anticancer activities of immune cells, inhibits immunosuppressive cells within the TME and finally exhibit enhanced inhibitory effects than any monotherapy. Moreover, current research also demonstrated the combined effects of IL-15 fusion protein with Nab-paclitaxel on colon cancer subcutaneous HCT116 model. IL-15 fusion protein binds to Nab-paclitaxel with high affinity to form a nanomedicine complex that has a cytotoxic and stimulating effect on colon cancer and immune cells, respectively. Flow cytometry results further demonstrated the enhanced accumulation and cytotoxicity for CD8^+^ T cells and NK cells, and decreased populations of Tregs and MDSCs. Further data also demonstrated that the enhanced anticancer immunity and decreased expression levels of immunosuppressive factors.

## 5. Conclusion

Combination therapy of Nab-paclitaxel and IL-15 fusion protein can effectively stimulate the antitumor activity of immune effector cells, thereby inhibiting immunosuppressive cells within the TME of colorectal cancer, and the overall therapeutic effect has a significant advantage over monotherapy.

## Highlight

- IL-15 fusion protein displayed the strong binding affinity for Nab-paclitaxel;
- IL-15 fusion protein enhanced antitumor efficacy of Nab-paclitaxel in HCT116 xenograft;
- IL-15 fusion protein potentiated anticancer immunity of Nab-paclitaxel in HCT116 xenograft;
- Nab-paclitaxel combined IL-15 fusion protein abated the NF-κB-mediated immunosuppression;
- Nab-paclitaxel combined IL-15 fusion protein enhanced apoptosis in HCT116 xenograft;

## References

[1] Wrobel P, Ahmed S. Current status of immunotherapy in metastatic colorectal cancer. Int J Colorectal Dis. 2019;34(1):13–25.3046523810.1007/s00384-018-3202-8

[2] Jin K, Ren C, Liu Y, et al. An update on colorectal cancer microenvironment, epigenetic and immunotherapy. Int Immunopharmacol. 2020;89(Pt A):107041.3304556110.1016/j.intimp.2020.107041

[3] Voutsadakis IA. The pluripotency network in colorectal cancer pathogenesis and prognosis: an update. Biomark Med. 2018;12(6):653–665.2994401710.2217/bmm-2017-0369

[4] Van der Jeught K, Xu H-C, Li Y-J, et al. Drug resistance and new therapies in colorectal cancer. World J Gastroenterol. 2018;24(34):3834–3848.3022877810.3748/wjg.v24.i34.3834PMC6141340

[5] Blondy S, David V, Verdier M, et al. 5-Fluorouracil resistance mechanisms in colorectal cancer: from classical pathways to promising processes. Cancer Sci. 2020;111(9):3142–3154.3253601210.1111/cas.14532PMC7469786

[6] Vodenkova S, Buchler T, Cervena K, et al. 5-fluorouracil and other fluoropyrimidines in colorectal cancer: past, present and future. Pharmacol Ther. 2020;206:107447.3175636310.1016/j.pharmthera.2019.107447

[7] Schmid P, Adams S, Rugo HS, et al. Atezolizumab and Nab-Paclitaxel in Advanced Triple-Negative Breast Cancer. N Engl J Med. 2018;379(22):2108–2121.3034590610.1056/NEJMoa1809615

[8] Yardley DA. nab-Paclitaxel mechanisms of action and delivery. J Control Release. 2013;170(3):365–372.2377000810.1016/j.jconrel.2013.05.041

[9] Glück S. nab-Paclitaxel for the treatment of aggressive metastatic breast cancer. Clin Breast Cancer. 2014;14(4):221–227.2480627810.1016/j.clbc.2014.02.001

[10] Yee NS. Update in Systemic and Targeted Therapies in Gastrointestinal Oncology. Biomedicines. 2018;6(1):34.10.3390/biomedicines6010034PMC587469129547556

[11] Galluzzi L, Chan TA, Kroemer G, et al. The hallmarks of successful anticancer immunotherapy. Sci Transl Med. 2018;10(459):eaat7807.3023222910.1126/scitranslmed.aat7807

[12] Pan C, Liu H, Robins E, et al. Next-generation immuno-oncology agents: current momentum shifts in cancer immunotherapy. J Hematol Oncol. 2020;13(1):29.3224549710.1186/s13045-020-00862-wPMC7119170

[13] Bagchi S, Yuan R, Engleman EG. Immune Checkpoint Inhibitors for the Treatment of Cancer: clinical Impact and Mechanisms of Response and Resistance. Annu Rev Pathol. 2021;16(1):223–249.3319722110.1146/annurev-pathol-042020-042741

[14] Katz H, Biglow L, Alsharedi M. Immune Checkpoint Inhibitors in Locally Advanced, Unresectable, and Metastatic Upper Gastrointestinal Malignancies. J Gastrointest Cancer. 2020;51(2):611–619.3102853710.1007/s12029-019-00243-8

[15] Sahin IH, Akce M, Alese O, et al. Immune checkpoint inhibitors for the treatment of MSI-H/MMR-D colorectal cancer and a perspective on resistance mechanisms. Br J Cancer. 2019;121(10):809–818.3160775110.1038/s41416-019-0599-yPMC6889302

[16] Yin Y, Yao S, Hu Y, et al. The Immune-microenvironment Confers Chemoresistance of Colorectal Cancer through Macrophage-Derived IL6. Clin Cancer Res. 2017;23(23):7375–7387.2892816110.1158/1078-0432.CCR-17-1283

[17] Hsu FT, Liu Y-C, Tsai C-L, et al. Preclinical Evaluation of Recombinant Human IL15 Protein Fused with Albumin Binding Domain on Anti-PD-L1 Immunotherapy Efficiency and Anti-Tumor Immunity in Colon Cancer and Melanoma. Cancers (Basel). 2021;13(8):1789.3391864110.3390/cancers13081789PMC8070266

[18] Weng MC, Li M-H, Chung JG, et al. Apoptosis induction and AKT/NF-κB inactivation are associated with regorafenib-inhibited tumor progression in non-small cell lung cancer in vitro and in vivo. Biomed Pharmacother. 2019;116:109032.3116338110.1016/j.biopha.2019.109032

[19] Voigt C, et al. Cancer cells induce interleukin-22 production from memory CD4(+) T cells via interleukin-1 to promote tumor growth. Proc Natl Acad Sci U S A. 2017;114(49):12994–12999.2915055410.1073/pnas.1705165114PMC5724250

[20] Hama M, Ishima Y, Chuang VTG, et al. Evidence for Delivery of Abraxane via a Denatured-Albumin Transport System. ACS Appl Mater Interfaces. 2021;13(17):19736–19744.3388129210.1021/acsami.1c03065

[21] Pham DT, Saelim N, Tiyaboonchai W. Paclitaxel loaded EDC-crosslinked fibroin nanoparticles: a potential approach for colon cancer treatment. Drug Deliv Transl Res. 2020;10(2):413–424.3170148810.1007/s13346-019-00682-7

[22] Hu T, Li Z, Gao C-Y, et al. Mechanisms of drug resistance in colon cancer and its therapeutic strategies. World J Gastroenterol. 2016;22(30):6876–6889.2757042410.3748/wjg.v22.i30.6876PMC4974586

[23] Kozovska Z, Gabrisova V, Kucerova L. Colon cancer: cancer stem cells markers, drug resistance and treatment. Biomed Pharmacother. 2014;68(8):911–916.2545878910.1016/j.biopha.2014.10.019

[24] Wu Z, Xu Y. IL-15R alpha-IgG1-Fc enhances IL-2 and IL-15 antitumor action through NK and CD8+ T cells proliferation and activation. J Mol Cell Biol. 2010;2(4):217–222.2067111610.1093/jmcb/mjq012

[25] Sun B, Hyun H, Li L-T, et al. Harnessing nanomedicine to overcome the immunosuppressive tumor microenvironment. Acta Pharmacol Sin. 2020;41(7):970–985.3242424010.1038/s41401-020-0424-4PMC7470849

[26] Pujade-Lauraine E, Wagner U, Aavall-Lundqvist E, et al. Pegylated liposomal Doxorubicin and Carboplatin compared with Paclitaxel and Carboplatin for patients with platinum-sensitive ovarian cancer in late relapse. J Clin Oncol. 2010;28(20):3323–3329.2049839510.1200/JCO.2009.25.7519

[27] Fabian KL, Storkus WJ. Immunotherapeutic Targeting of Tumor-Associated Blood Vessels. Adv Exp Med Biol. 2017;1036:191–211.2927547310.1007/978-3-319-67577-0_13

[28] Chen DS, Mellman I. Oncology meets immunology: the cancer-immunity cycle. Immunity. 2013;39(1):1–10.2389005910.1016/j.immuni.2013.07.012

[29] Waldmann TA, Dubois S, Miljkovic MD, et al. IL-15 in the Combination Immunotherapy of Cancer. Front Immunol. 2020;11:868.3250881810.3389/fimmu.2020.00868PMC7248178

[30] Hinrichs CS. Can interleukin-15 keep its therapeutic promise? Sci Transl Med. 2018;10(431):eaar7532.

[31] Conlon KC, Lugli E, Welles HC, et al. Redistribution, hyperproliferation, activation of natural killer cells and CD8 T cells, and cytokine production during first-in-human clinical trial of recombinant human interleukin-15 in patients with cancer. J Clin Oncol. 2015;33(1):74–82.2540320910.1200/JCO.2014.57.3329PMC4268254

[32] Wrangle JM, Velcheti V, Patel MR, et al. ALT-803, an IL-15 superagonist, in combination with nivolumab in patients with metastatic non-small cell lung cancer: a non-randomised, open-label, phase 1b trial. Lancet Oncol. 2018;19(5):694–704.2962831210.1016/S1470-2045(18)30148-7PMC6089612

